# Chemical Composition, Antioxidant, Insecticidal Activity, and Comparative Analysis of Essential Oils of Leaves and Fruits of *Schinus molle* and *Schinus terebinthifolius*

**DOI:** 10.1155/2022/4288890

**Published:** 2022-05-30

**Authors:** Oumayma Belhoussaine, Chaimae El Kourchi, Hicham Harhar, Abdelhakim Bouyahya, Adil El Yadini, Fozia Fozia, Amal Alotaibi, Riaz Ullah, Mohamed Tabyaoui

**Affiliations:** ^1^Laboratory of Materials, Nanotechnology and Environment, Faculty of Sciences, Mohammed V University in Rabat, Av. Ibn Battouta, B. P 1014, Rabat, Morocco; ^2^Laboratory of Human Pathologies Biology, Department of Biology, Faculty of Sciences, Mohammed V University in Rabat, Rabat, Morocco; ^3^Biochemistry Department, Khyber Medical University Institute of Medical Sciences, Kohat, Khyber Pakhtunkhwa, Pakistan; ^4^Department of Basic Science, College of Medicine, Princess Nourah Bint Abdulrahman University, P.O. Box 84428, Riyadh 11671, Saudi Arabia; ^5^Department of Pharmacognosy (MAPPRC), College of Pharmacy, King Saud University, Riyadh 11451, Saudi Arabia

## Abstract

*Schinus terebinthifolius* Raddi. and *Schinus molle* L. are perennial woody plants belonging to the Anacardiaceae family, widely distributed in the United States, Europe, Asia, and Africa, and they are broadly used for many applications such as in traditional medicine as an antipyretic, analgesic, depurative, and in the treatment of diseases of the urogenital system as well as culinary and ornamental species. Our work aims to study and compare the chemical composition and the antioxidant and insecticidal activity of the essential oils of the leaves and fruits of the two species of the genus *Schinus*. The essential oils were characterized by a very spicy aromatic odor, and by the abundance of hydrocarbon monoterpenes in the leaves and fruits of *Schinus molle* (49.70% and 42.65%), unlike the EOs of the fruits of *Schinus terebinthifolius* which have a high content in hydrocarbon sesquiterpenes (40.57%). Usually, these oils have shown relatively low antioxidant activity was expressed in IC_50_; especially, the essential oil of the fruits of *S. terebinthifolius* revealed a concentration of 3.292 ± 2.82 mg/mL. The evaluation of the insecticidal activity gave good results in the method of exposure of adults of *Sitophilus oryzae* to EOs by contact; thus, the fruits of *Schinus molle* are more active against this species of beetle than the other essential oil.

## 1. Introduction

The family Anacardiaceae has about 60 to 74 genera and 400 to 600 species. The Anacardiaceae consists of trees, shrubs, lianas, or rarely perennial herbs and tissues of plant organs with resinous conduits or laticifers [1, 2]. The genus *Schinus* has about 30 species, most of which are found in a spontaneous state in the South American region [3]. *Schinus molle* L. and *Schinus terebinthifolius* Raddi. are known by various common names such as false pepper, Brazilian pepper, and *Aroeira* and are native to Brazil and introduced in several countries of the world [4–6].

*Schinus molle* L. (S.M.) is commonly known as “aguaribay,” “bálsamo,” “chichita,” “Gualeguay,” “molle,” “pimentero,” and “erebinto,” a sparsely cultivated wild plant that can grow up to 25 m tall but 0.5 to 1.5 m in diameter at the base [1]. The fruits of *S. molle* are commercialized under the name of pepper (pink pepper), much appreciated in the Mediterranean cuisine [7]. Leaves composed of 3 to 10 pairs of leaflets, with serrated edges. When it blooms, from September to January, its small aromatic flowers, light yellow in color, attract bees. The flowers are unisexual, hermaphrodite, and arranged in elongated panicles. The fruits are globular drupes of 4 to 6 mm of diameter, round, red, and brilliant and gathered in hanging clusters. *Schinus molle* and *S. terebinthifolius* were used to treat urinary tract infections, skin ulcers, gastroduodenal disorders, and ulcers and infections of the respiratory, digestive, and genitourinary systems. *Schinus molle* is also taken as a diuretic and a digestive tonic for cleansing the system. It presents red and edible pulp [8]. The essential oil (EO) of leaves and fruits of Brazilian *S. molle* contains as major compounds sabinene (48.63% and 51.74%) and limonene (10.20% and 16.98%), respectively, while bicyclogermacrene (18.12%) was also important in the leaf oil [9]. Previous studies have reported that the EOs of *S. molle.* are characterized by their antioxidant, antimicrobial [10–14], cytotoxicity, and insecticidal proprieties [3, 14–16].

*Schinus terebinthifolius Raddi* (*S. terebinthifolius*), called “*aroeira-vermelha*,” “*aroeira-pimenteira*,” “Brazilian pepper,” Christmas berry, pink pepper [5], is a dioecious tree of medium size, with a short trunk, generally hidden by interlaced branches. It reaches a height of 5 to 10 meters. Its leaves are dark green and oblong to elliptical. The white or yellow flowers are small and grouped in bouquet-like inflorescences. The bark of the *Schinus* has an action against fever, hemoptysis, and uterine disorders in general. From the shell, oil is used to treat tumors and diseases of the cornea [17]. *S. terebinthifolius* was also widely used in Brazilian traditional medicine for many purposes as an anti-inflammatory and healing and to treat some respiratory diseases [6]. In fact, some recent in vitro and in vivo studies [18] have reported numerous biological activities of *S. terebinthifolius* extracts such as antioxidant, antibacterial, and antifungal [19, 20]. The essential oils of the leaves and fruits are rich in limonene (14.21–16.99%), germacrene D (11.45–10.85%), and cadinene (9.21–3.31%), respectively [17].

*Sitophilus oryzae* L. (*S. oryzae*) (Coleoptera: Curculionidae), a ubiquitous pest of economic importance, is an internal feeding insect that burrows into the stored grain. Adult weevils feed primarily on endosperm, which reduces carbohydrate content, and the larvae preferentially feed on the germ of the grain, removing much of the protein and vitamins. Insects that selectively attack the germ will cause greater loss of germination than others [21].

The aim of this study was to evaluate the chemical composition of *S. molle* and *S. terebinthifolius* leaf and fruit essential oils by GC-MS, antioxidant properties by DPPH free radical scavenging method, and insecticidal activity by contact, repellency, and fumigation against wheat weevil (*S. oryzae*).

## 2. Materials and Methods

### 2.1. Preparation of Plant

The leaves and fruits of both species of *Schinus* were collected from the region of Rabat (34°01′53.34″) in the month of February-March. The confirmation of both species was carried out by Prof. El Aboudi Ahmed, a botanist at the department of Biology, Faculty of Sciences Mohammed V University. The two parts of the plants were separated and dried away from humidity after two weeks and then crushed in order to perform the extraction.

### 2.2. Extraction of Essential Oil

The extraction of essential oils by hydrodistillation of *S. molle* and *S. terebinthifolius* was achieved using a Clevenger-type instrument [22]. First, 100 g of crushed leaves or fruits of *S. molle* and *S. Terebinthifolius* was placed in a 1000 ml flask at a plant material/water ratio of 1 : 3. The flask was heated for 6 h. The extraction was continued until no essential oil was collected. The resulting mixture of water and essential oils was then dehydrated and stored in dark bottles.

### 2.3. Chemical Analysis of Essential Oils by GC-MS

Analyses were carried out using a Perkin-Elmer Clarus 690 (Waltham, MA, USA) equipped with dual flame ionisation detection (FID) system and fused-silica capillary columns, namely, Rtx-1 (polydimethylsiloxane) and Rtx-wax (poly-ethyleneglycol) (60 m × 0.25 mm i. d; film thickness 0.25 *μ*m). The oven temperature was programmed from 60 to 230°C at 2°C/min and then held isothermally at 230°C for 30 min: hydrogen was employed as carrier gas (0.7 mL/min). The injector and detector temperatures were maintained at 280°C, and samples were injected (0.5 *μ*L HE diluted in ethanol grade FID) in the split mode (1/80). Retention indices (RI) of compounds were determined relative to the retention times of a series of n-alkanes (C5C30) by linear interpolation using the Van den Dool and Kratz equation with the aid of software from Perkin-Elmer (Total Chrom navigator). The relative percentages of the oil constituents were calculated from the GC peak areas, without the application of correction factors.

Samples were also analysed with a gas chromatograph of the Hewlett-Packard type (HP 6890 series) coupled with a mass spectrometer (HP 5973 series). Fragmentation is carried out by electronic impact under a field of 70 eV. The column used is an HP-5 MS capillary column (30 m x 0.25 mm), and the film thickness is 0.25 *μ*m. The temperature of the column is programmed from 50 to 250°C at a rate of 4°C/min. The carrier gas is helium, the flow rate of which is set at 1.5 mL/min. The injection mode is split (leakage ratio: 1/70, flow rate 112 mL/min). The device is connected to a computer system managing a NIST 11 mass spectrum library.

### 2.4. Evaluation of Antioxidant Activity

The antioxidant power of the essential oils of the four samples was tested by the DPPH (2,2-diphenyl picryl-hydrazyl) as a relatively stable free radical method [23]. The reaction is achieved in a total volume of 2.5 ml containing 0.5 ml of DPPH at 0.2 mM solubilized in methanol. The essential oil samples were prepared by dissolving in absolute methanol at 20 mg/ml, and these solutions will then be diluted to obtain the final concentrations of 15%, 17.5%, 20%, 22.5%, and 25% in *S. molle* and *S. terebinthifolius* fruits and concentrations of 25%, 50%, 75%, and 100% for *S. molle* and *S. terebinthifolius* leaves. For each concentration, the test is repeated twice. The samples are then left in the dark for 30 minutes, and the discoloration compared to the negative control containing only the DPPH solution is measured at 517 nm using a UV spectrometer. The antioxidant activity is estimated according to the following equation [24]:

(1) $$\begin{array}{c} \text{AA}\%=\left[\frac{\left(\text{Abs control}-\text{Abs test}\right)}{\text{Abs control}}\right]\times 100, \end{array}$$

- Abs control is the absorbance of the negative control,
- Abs test is the absorbance of the tested compound.

### 2.5. Insecticidal Activity

#### 2.5.1. Mass Breeding

A quantity of rice contaminated with *S. Oryzae* is added to tightly closed jars containing healthy rice. These jars were left for one month at room temperature until the emergence of adults. The objective of this breeding is to produce a sufficient mass of individuals.

#### 2.5.2. Assessment of Insecticidal Activity by Contact

The contact toxicity of extracted EOs for adults of *S. Oryzae* was evaluated in acetone to obtain the required concentrations. About 25 to 200 *μ*L of EO was applied to the surface. The oil + acetone solution is uniformly distributed on a disc of filter paper, and a control receives 200 *μ*L of acetone only. Four adults of *S. Oryzae*, individuals are placed on the filter paper in the middle of the Petri dishes (5.5 cm diameter × 1.5 cm). Mortality control was carried out by counting dead insects from the first day of treatment until the death of all individuals [25].

#### 2.5.3. Assessment of Insecticidal Activity by Fumigation

The fumigant effect of EOs was determined according to the method of Khani and Asghari [26], with some modifications. Four adults of *S. Oryzae* were placed in 50 mL plastic bottles. 5, 25, 50, 100, and 150 *μ*L of EO were added to individual 3 cm diameter filter paper. The filter paper was then attached to the undersurface of the cap firmly attached to the vial to produce concentrations of 0.1, 0.5, 1, 2, and 3 *μ*L/L air, respectively. The control vial did not receive any trace of oil. Insect mortality was determined after 24, 48, 72, 96, 120, 144, 168, and 192 hours of exposure. Insects were considered dead when they could no longer move parts of their bodies.

#### 2.5.4. Repellent Activity

The study of the repulsive power of the EOs was achieved by calculating the percentage of repulsion of the studied EOs towards *S. Oryzae* by the preferential area method on filter paper described by Jilani and Saxena [27]. Filter paper discs of 11 cm diameter are cut into two equal parts; one half of the paper is treated with EOs plus acetone, and the other half is treated with acetone only. 25, 50, 100, 150, and 200 *μ*L of essential oil are diluted, respectively, in 200 *μ*L of acetone so that the distribution is homogeneous on the filter paper. Four insects were introduced in the middle of the Petri dishes. The solution (oil + acetone) is evenly distributed on one half of the filter paper disc, and the other half of the disc receives acetone only. The two half discs of filter paper are air-dried, and the disc is reconstituted and put in a Petri dish. After half an hour of treatment of the insects under laboratory conditions, the count of the insects on the half disks is achieved. The percentage of repulsion (PR) is thus calculated according to the formula used by Nerio et al. [28] as follows:

(2) $$\begin{array}{c} \text{Repellency}\%=\left[\frac{\left(N_{\text{ac}}-N_{\text{EO}}\right)}{\left(N_{\text{ac}}+N_{\text{EO}}\right)}\right]*100, \end{array}$$

- *N*_ac_ : Number of insects present on the half disc treated with acetone,
- *N*_EO:_ Number of insects present on the half disc treated with the oil solution.

## 3. Results and Discussion

### 3.1. Essential Oil Yield

The essential oil obtained from *S. molle* is pale yellow color contrary to the oil of *S. terebinthifolius* which is of greenish yellow color, with a very spicy peppery aromatic smell in both species.

The yield of essential oil from the leaves and fruits of each of the two species is expressed in percentage and is presented in Table 1.

The determination of the yield according to the used parts of the plant detected a difference in yield between the leaves and fruits of *S. terebinthifolius*. Otherwise, the determination of the yield according to the selected plant revealed that *S. molle* is richer in essential oil than *S. terebinthifolius.*

A study carried out by Santos et al. [9] on the extraction of Brazilian *S. molle* leaves and fruits, and *S. terebinthifolius* leaves and fruits by a Clevenger apparatus and during 1 h of distillation, gave a yield of 1.24% and 0.49% for the leaves and fruits, respectively, for S.M., while for S.T., the yield is 0.74% and 0.16%, respectively.

In 2012, Santana et al. [29] found that the EO content of *S. terebinthifolius* leaves is around 0.17%. In Costa Rica, Martins et al. [30] reported that *S. molle* leaves are very rich in EO than fruits, with a content of 1.09% and 0.91%, respectively. Dos Santos Cavalcanti et al. [31] achieved the extraction of 80 g each of the leaves and fruits of *S. molle* and *S. terebinthifolius* by hydrodistillation for 6 h and found that the EO content is very low in the leaves of *S. terebinthifolius* of about 0.10%, while the content of fruits is 1.74% and the EO yield in *S. molle* is very high in fruits than in leaves of about 2.30% and 1.10%, respectively, which remains much lower than our results around 2%.

### 3.2. Chemical Composition

GC-MS analysis showed a difference in the chemical composition of the EOs of the two species studied. A total of 46 and 44 components were identified in *S. molle* and *S. terebinthifolius* representing, respectively, for leaves-Fruits (91%-92%) and (89%–84%) of the total content given in Table 2.

The EO of *S. molle* is characterized by the presence of *γ*-muurolene, *γ*-gurjunene, *γ*-cadinene, 10-epi-elemol, guaiol, and *α*-acorenol, while that of *S. terebinthifolius* can be distinguished by the presence of *β*-gurjunene and the absence of the compounds mentioned above. The majority of the compounds present in the essential oil of *S. molle* (leaves and fruits) are *β*-pinene (10.36–5.44%), *γ*-terpinene (12.01–8.15%), limonene (22.94–18.49%), 10-epi-elemol (7.64–8.03%), *γ*-eudesmol (5.17–4.09%), and longifolene (7.67–8.48%). And those present in the EO of *S. terebinthifolius* (leaves and fruits) are *γ*-terpinene (9.45–6.70%), limonene (23.22–6.52%), spathulenol (14.34–6.84%), *β*-ocimene (13.32–0%), sabinol (5.07% and —), germacrene D (2–8.53%), *γ*-elemene (0.42–10.11%), *γ*-eudesmol (— and 3.59%), *τ*-muurolol (— and 3.46%), and longifolene (— and 3.51%). *β*-myrcene, *γ*-terpinene, limonene, longifolene, and *γ*-eudesemol are the majority compounds identified in the four essential oils, while spathumenol is determined only in the extracts of ST, and 10-epi-elemo characterizes those of SM.

The fruits of ST are particularly characterized by the presence of the molecules: globulol, *γ*-elemene, and *β*-elemene, or the leaves obtain the sabinol and those of SM mark the presence of *β*-ocimene.

The essential oils of the leaves of *S. molle* and *S. terebinthifolius* are predominated by monoterpene compounds (56.25% and 67.51%), while those of the fruits are characterized by the presence of sesquiterpene compounds (45.90% and 57.99%). Structures of the majority of compounds identified in the two *Schinus* species are given in Figure 1.

The chemical group composition of *S. molle* and *S. terebinthifolius* essential oil (peak area %) is given in Figure 2. The hydrocarbon monoterpenes present the majority constituents of the EO of the leaves and fruits, respectively, of *S. molle* (49.70% and 42.65%), while in *S. terebinthifolius*, the chemical composition differs between the parts used of the plant where we find that the leaves are rich in hydrocarbon monoterpenic compounds 55.69% contrary to the fruits which are dominated by hydrocarbon sesquiterpenes 40.57%.

Previous studies that have been achieved on the EOs of both species stated that these oils are rich in monoterpene compounds, which is compatible with our results, but the difference lies in the dominant monoterpene compounds which differ from one study to another. However, Bendaoud et al. [32] stated that the main difference between the essential oils of the genus *Schinus* is the high content of sesquiterpenes in the fruits of *S. terebinthifolius* which is similar to our results.

The chemical composition of essential oils of *S. molle* marks a difference with that collected in Tunisia, and this fruit oil is characterized by a high percentage of hydrocarbon monoterpenes 79.69% and 11.75% of oxygenated monoterpenes with only 3.69% of hydrocarbon sesquiterpenes and 1.83% oxygenated sesquiterpenes. Specifically, this oil showed high content of *α*-phellandrene (46.52%) and *β*-phellandrene (20.81%) [32]. Eryigit et al. [33] found that *S. molle* fruits grown in Turkey yield EO rich in *α* and *β*-phellandrene (31.74 and 16.49%) and p-cymene (11.36%). Also, Aboalhaija et al. [34] compared the EOs of leaves and fruits from different regions of Jordan and marked that stereoisomers *α*- and *β*-phellandrene represent the major components of the EOs studied, while the essential oil of *S. molle* fruits grown in Mexico gave a high percentage of myrcene (39.7), p-cymene (19.5%), cadinene (7.8%), and phellandrene (7.1%) [35].

We found a significant difference in the chemical composition of the EOs of *S. terebinthifolius*. However, the oil of the leaves collected from the north of Brazil recorded major compounds different from what we obtained such as p-cymen-7-ol (22.5%), 9-epi-(E)-caryophyllene (10.1%), carvone (7.5%), and verbenone (7.4%) [36]. However, fruits collected by Do Nascimento et al. [37] in Brazil have as major compounds thujene (21.7%), sabinene (15.8%), *α*-phellandrene (11.9%), and limonene (31.8%). From the same region, Dos Santos Cavalcanti et al. [31] compared the chemical composition of *S. terebinthifolius* EOs and found that leaves are characterized by the abundance of tricyclene (8.3%), eucalyptol (8.5%), and *β*-caryophyllene (35.2%), while fruits are distinguished by the presence of oxygenated sesquiterpene compounds that are absent in leaves.

### 3.3. Antioxidant Activity

In vitro antioxidant activity test was carried out by varying the concentration of the methanolic extracts of essential oils studied by calculating the inhibitor percentage for each concentration from the absorbance obtained by spectrometry at 517 nm. The results are grouped into two graphs (Figures 3(a) and 3(b)), one to compare the percentages of inhibition of EOs of the fruits and the other of the leaves of both species.

The evaluation of the antioxidant activity of the EO of leaves and fruits (5 mg/mL) revealed a percentage of radical inhibition of 17.99% and 53.30% in *S. molle* and 49.31% and 77.82% in *S. terebinthifolius*, respectively, which shows that the fruits exhibited higher antioxidant activity than the leaves.

The antioxidant effect of the different EOs was expressed in IC_50_, which represents the 50% inhibitory concentration of the radicals with reference to ascorbic acid (Table 3).

The calculation of the IC_50_ of the 4 oils studied showed that they have a rather low antioxidant activity compared to the reference antioxidant. However, comparing the IC_50_ of the essential oils of leaves and fruits, we find that fruits have a higher activity than leaves, and this may be due to the richness of the berries by sesquiterpene compounds (hydrocarbon and oxygenated). However, the essential oil of the fruits of *S. terebinthifolius* revealed a concentration of 3.292 ± 2.82 mg/mL higher than that of ascorbic acid (1.91 *μ*g/mL) and lower than those of other EOs, which proves that *S. terebinthifolius* fruits have a stronger antioxidant activity than *S. molle fruits*, and this can be attributed to the presence of globulol characterizing the fruits of *S. terebinthifolius*.

In the literature, the essential oils of *S. molle* leaves and fruits have reported low antioxidant activity [30, 38, 39]. These authors correlated their results with the small percentage of oxygenated terpene.

In summary, the chemical composition of EOs is responsible for this low antioxidant activity due to the fact that monoterpenes present the majority of the components of these EOs. This has been reported by several authors [40–43], who stated that essential oils rich in monoterpenes such as *α*-pinene, *β*-pinene, limonene, *β*-myrcene, sabinene, and terpinolene did not show strong antioxidant activities.

### 3.4. Insecticidal Activity

#### 3.4.1. Assessment of Insecticidal Activity by Contact

Evaluation of contact insecticidal activity showed that insect mortality increased with increasing concentrations of 0–200 *μ*L/cm^2^ and duration of exposure to essential oils (Figures 4 (a)–4(d)). The lowest mortality values are recorded in the control boxes; they are 25% after 7 days of exposure. The EOs used at doses of 200, 150, and 100 *μ*L/cm^2^ showed higher mortality rates and even from the first day in the fruit EOs of the two species studied.

The essential oil of *S. molle* fruits reported 100% mortality against *S. oryzae* at 25 *μ*L/cm^2^ concentration after 3 days of exposure, while for leaves, this mortality value was marked after 7 days of exposure for the same concentration. Thus, Petri dishes of 200 *μ*L/cm^2^ concentration recorded a mortality rate of 100% after the first and second day of exposure for fruits and leaves, respectively.

For the essential oil of *S. terebinthifolius*, a mortality rate of 100% was reached at a concentration of 25 *μ*L/cm^2^ after 8 days of exposure for fruits and leaves. While at a concentration of 200 *μ*L/cm^2^, the boxes record the total mortality of the insects after 1 and 2 days of exposure to the essential oils of fruits and leaves, respectively.

The evaluation of the insecticidal activity of the EO of the leaves and fruits of the two species showed a significant difference based on the calculation of the lethal dose 50 (LD_50_) which represents the concentration marking 50% of the mortality of insects (Table 4).

The lethal dose 50 (LD_50_) was determined graphically from the plots representing the mortality rates after 24 h of exposure of insects to essential oils as a function of concentrations and is presented in Table 4.

In the light of these results, the EO of the fruits of *S. molle* has a higher insecticidal activity due to the fact that its lethal dose (50 *μ*L/cm^2^) is lower than that of the leaves contrary to *S. terebinthifolius* which showed a lower lethal dose in leaves (83.33 *μ*L/cm^2^) than in fruits, while Mohamed and Abdelgaleil [44] found that the essential oil of *S. terebinthifolius* leaves used for contact treatment on *S. oryzae* marks an LD_50_ = 0.42 mg/cm^2^.

The analysis of the insecticidal effect of the EOs of the false pepper tree revealed significant differences for the factors oils, doses, and duration of exposure, which made it possible to classify the oils used according to their toxicities. The DL_50_ decreases with increasing duration of EO exposure, and we find that SMF is the most toxic (Figure 5).

The essential oil of *S. molle* fruits represents 50% mortality at a concentration of 50 *μ*L/cm^2^, and this may be due to its special chemical composition characterized by the presence of *β*-linalool (0.23%), thujone (0.34%), and ledol (0.36%). However, Mohamed and Abdelgaleil [44] stated that alcoholic monoterpenes such as geraniol, linalool, and menthol have a pronounced activity on *S. oryzae*. Park et al. [45] stated that the essential oil of *Chamaecyparis obtusa*, in a toxicity study against adults of *S. oryzae* exposed to direct contact, gave 80% mortality at 0.26 mg/cm^2^ due to the presence of bornyl acetate and terpinolene.

#### 3.4.2. Assessment of Insecticidal Activity by Fumigation

Assessment of the insecticidal activity of *S. molle* and *S. terebinthifolius* essential oils by fumigation on *S. oryzae* adults showed that these oils are less effective against these insects by comparing their contact activities (Figure 6). In the treated batches, Weevil death ranged from 2 to 7 days, whereas in the control batch, this parameter ranged over 7 days. Thus, the toxicity of EOs depends on the dose and duration of exposure. The death of insects increases as the dose and the exposure time increase.

The batches of 5 *μ*L/L of air recorded a mortality rate of 75% and 50% after 8 days of exposure to the essential oils of the fruits and leaves, respectively, of *S. molle*, while the batches of 150 *μ*L/L of air marked a mortality rate of 100% after 5 and 4 days of exposure to the EOs of the fruits and leaves of SM (Figures 6(a) and 6(b)).

The batches of 5 *μ*L/L of air did not record any mortality after 8 days of inhalation of essential oils of the leaves and fruits of S.T. which explains the low activity of this plant on *S. oryzae*, while the batches of 150 *μ*L/L of air marked a mortality rate of 100% and 75% after 7 days of inhalation with essential oils of fruits and leaves, respectively, of *Aroeira* (Figures 6(c) and 6(d)).

Mohamed and Abdelgaleil [44] tested the fumigant effect of *S. terebinthifolius* and revealed LC_50_ = 56, 48 *μ*L/L air after 72 h of exposure, which reveals that it has a moderate fumigant activity compared to *Mentha microphylla* which is very strong. Sahaf et al. [46] found that the highest concentration of *Vitex pseudo-negundo* oil (925.9 *μ*L/L air) induces more than 50% mortality after 6 h and reached a level of 100% at 12 h after treatment. The lowest concentration was found to be capable of killing 50% of *S. oryzae* within 24 h. At 740.7 *μ*L/L of air, complete mortality of beetles was achieved after 15 h of exposure. Moreover, Negahban et al. [47] found that the essential oil of *Artemisia siberi* has a good fumigant activity against *S. oryzae* by registering 50% mortality at a concentration of 3.86 *μ*L/L air. Alternatively, Benzi et al. [48] tested the insecticidal activity of EOs from the leaves and fruits of *S. molle* on *S. oryzae* and reported that these did not produce a fumigant effect on *S. oryzae* adults during the 4 days tested, and this may have been due to the fact that the entry of these compounds is through the cuticle and has higher concentrations to achieve mortality or to a longer exposure time. According to Pérez-López et al. [35], rice weevils are sensitive to coriander essential oil with a percentage of mortality equal to 56% in 24 h.

#### 3.4.3. Repellency activity

The repellent activity of the studied EOs, after an exposure time of 30 min, is dependent on the dose deposited in the Petri dishes. This activity increases as the dose increases, and it also depends on the used part of the plant (Figure 7).

For berries, it can be seen that *S. molle* is highly repellent to adults of *S. oryzae* than *S. terebinthifolius* which is moderately repellent even at the highest dose. Thus, at the dose of 150 *μ*L/cm^2^, both plants are moderately repellent, whereas at 100 *μ*L/cm^2^ and 50 *μ*L/cm^2^, *S. molle* alone has a repellent activity.

For leaves, *S. molle* is more repellent than *S. terebinthifolius* at 200 *μ*L/cm^2^ and 150 *μ*L/cm^2^ doses, while at 100 *μ*L/cm^2^, they have the same percentage of repellency.

The calculation of the average percentage of repulsion of different doses by the method of McDonald et al. [49] shows that the EO of fruits *S. molle* and *S. terebinthifolius* and *S. molle* leaves is moderately repulsive and belongs to class II with percentages of 28.18%, 26.66%, and 21.52%, respectively, while that of *S. terebinthifolius* leaves is weakly repellent (8.56%) and belongs to class I. The probit analysis showed that *S. oryzae* was more sensitive (RD_50_ = 0.084 *μ*L/cm^2^) to coriander EO than linalool standards (RD_50_ = 0.206 *μ*L/cm^2^) according to Sriti Eljazi et al. [50]. Therefore, it is important to explore the uses of medicinal plants because they are used for the treatment of different infections. World Health Organization reports that various plant fractions and their dynamic constituents are utilized as traditional medicines by 80% of the world population [51–54].

## 4. Conclusion

Loss of cereals caused by insect pests remains a problem of concern to farmers through reduction in commercial value and viability of seeds. However, the use of plants to fight against these beetles has become a famous objective. In our study, the insecticidal and antioxidant activity of EOs of the two species of the genus *Schinus* against *S. oryzae* was explored. The comparative study of these species allowed noticing the insecticidal effect of the fruits against *S. oryzae*, so the chemical analysis shows the presence of different constituents responsible for this insecticidal activity. However, the abundance of monoterpenes is accompanied by a weak antioxidant activity of essential oils. Finally, we can conclude that the fruits of *S. molle* can be used for the preservation of stored foodstuffs.

## Figures and Tables

**Figure 1:** Structures of the majority compounds identified in the two *Schinus* species.

**Figure 2:** Chemical group composition of *S. molle* and *S. terebinthifolius* essential oil (peak area %).

**Figure 3:** (a, b) Percentage of radical inhibition (% RSA) of the different essential oils studied.

**Figure 4:** Mortality rate of *Sitophilus oryzae* treated with different essential oils by contact. (a) SMF; (b) SML; (c) STF; (d): STL.

**Figure 5:** Lethal dose (DL_50_) of different essential oils according to exposure days.

**Figure 6:** (a–d) Mortality rate of *S. oryzae* adults treated by fumigation with EOs from *S. molle* (a, b) and *S. terebinthifolius* (c, d).

**Figure 7:** Repellency % of fruits and leaves essential oils of *Schinus molle* (SMF and SML) and *Schinus terebinthifolius* (STF and STL).

**Table 1:** Yields of different essential oil of *S. molle* and *S. terebinthifolius*.

	*Schinus molle*		*Schinus terebinthifolius*	
	SML	SMF	STL	STF
Yield%	2.97 ± 0.02	2.67 ± 0.02	0.28 ± 0.01	2.14 ± 0.04

*Note*. SML: Essential oil of leaves of *Schinus molle*; SMF: essential oil of fruits of *Schinus molle*; STL: essential oil of leaves of *Schinus terebinthifolius*; STF: essential oil of fruits of *Schinus terebinthifolius.* Extractions are repeated three times.

**Table 2:** Chemical composition of different essential oils.

Compound name	Retention indices		*Schinus molle*		*Schinus terebinthifolius*	
	RI I	RI a	SML	SMF	STL	STF
*α*-Pinene	936	934	—	**0.70**	—	**3.26**
Camphene	950	948	**0.21**	**2.22**	**0.91**	—
*β*-Pinene	978	974.96	**0.24**	**1.21**	**1.48**	**0.25**
*β*-Myrcene	987	983	**10.36**	**5.44**	**4.22**	**0.70**
(+)-2-Carene	996	996	**3.19**	—	—	—
*α*-Phellandrene	998	1001	**0.22**	**0.75**	**0.96**	—
*α*-Terpinene	1013	1014	**12.01**	**8.15**	**9.45**	**6.70**
Limonene	1025	1026	**22.94**	**18.49**	**23.22**	**6.52**
*β*-Ocimene	1027	1028	—	**5.04**	**13.32**	—
*γ*-Terpinene	1051	1052	**12.01**	**8.15**	**9.45**	**6.70**
Terpinolene	1086	1082	**0.50**	**0.61**	**2.09**	**0.77**
Linalool	1086	1085.36	—	**0.23**	—	—
*α*-Thujone	1087	1089	—	**0.34**	—	—
*α*-Campholenal	1105	1110	—	—	**0.20**	—
Sabinol	1120	1121	**2.52**	**1.57**	**5.07**	**0.33**
Trans-p-menth-2-en-1-ol	1123	1127	**0.75**	—	**0.62**	—
Octanoic acid methyl ester	1125	1126	**2.26**	—	—	—
Verbenol	1128	1130	—	—	**0.28**	—
Para-cymen-8-ol	1162	1163	**0.28**	—	**0.77**	—
Terpinen-4-ol	1164	1165.28	**0.44**	**0.36**	**0.37**	—
Pinocarveol	1184	1187	—	—	**0.40**	—
Carvone	1214	1219	—	—	**0.27**	—
Piperitone	1232	1231	—	—	**0.35**	—
Carvenone	1236	1234	**0.89**	**0.24**	**1.26**	—
Phellandral	1249	1250	**0.30**	—	**0.42**	—
Thymol	1267	1278	**1.33**	**0.82**	**1.75**	—
Bornyle acetate	1273	1279	**0.29**	**0.52**	—	—
Carvacrol	1278	1286	—	—	—	**0.37**
Citronellol acetate	1334	1337	—	—	**2.25**	—
Geranyl acetate	1358	1357	**0.30**	—	**0.50**	—
*β*-Elemene	1389	1389.71	**0.47**	**1.39**	**0.26**	**8.15**
*α*-bisabolol	1665	1666	**0.61**	—	—	—
Caryophyllene oxide	1578	1573	—	**0.34**	**0.28**	**0.22**
*α*-gurjunene	1409	1410	**0.27**	**0.65**	—	**0.21**
Longifolene	1411	1412	**7.67**	**8.48**	—	**3.51**
Caryophyllene	1421	1423.55	**1.16**	**1.03**	**0.41**	**3.75**
*β*-gurjunene	1424	1425	—	—	**0.53**	**0.50**
*α*-humulene	1451	1453	**0.34**	**0.64**	—	**0.47**
Alloaromadendrene	1462	1461.15	—	**0.77**	**0.66**	**2.67**
*γ*-gurjunene	1475	1473	**0.25**	**2.07**	—	—
Germacrene D	1479	1479.72	**0.62**	**1.40**	**2.00**	**8.53**
Géranyl isobutyrate	1484	1486	**2.03**	—	—	—
Amorphene	1490	1491	—	**0.31**	—	—
*α*-muurolene	1496	1495.87	**0.63**	—	—	—
*γ*-cadinene	1507	1508	**0.40**	**0.70**	—	—
*δ*-cadinene	1520	1518.13	**1.97**	**3.47**	**0.35**	**1.90**
*α*-calacorene	1528	1529	—	—	—	**0.24**
Sélina-3,7 (11)-diene	1539	1540	—	—	—	**0.49**
Spathulenol	1572	1570.65	**0.88**	**3.69**	**14.34**	—
Globulol	1579	1576	—	—	—	**5.13**
Viridiflorol	1580	1581	**0.33**	**0.76**	—	**2.78**
Guaiol	1582	1584	**0.74**	**1.06**	—	—
Ledol	1586	1597	—	**0.36**	—	—
*α*-acorenol	1616	1614	**0.54**	**0.80**	—	—
*γ*-eudesmol	1618	1620	**5.17**	**4.09**	—	**3.59**
*τ*-muurolol	1632	1641.01	—	**2.78**	—	**3.46**
*β*-eudesmol	1641	1633	—	—	—	**0.490**
*γ*-elemene	1727	1725	—	**2.37**	**0.42**	**10.11**
10-epi-elemol	2141	2142	**7.64**	**8.03**	—	—

**Table 3:** IC_50_ of different essential oil of *S. molle* and *S. terebinthifolius*.

	*Schinus molle*		*Schinus terebinthifolius*		Ascorbic acid
	SML	SMF	STL	STF	
IC_50_ (mg/mL)	10.100 ± 1.19	4.134 ± 0.41	8.680 ± 7.57	3.292 ± 2.82	0.00191

**Table 4:** The lethal dose 50 of the different essential oils studied.

	*Schinus molle*		*Schinus terebinthifolius*	
	SML	SMF	STL	STF
LD_50_ (*μ*L/cm^2^)	100 ± 0.000	50 ± 0.001	83.33 ± 0.014	100 ± 0.000

## Data Availability

All the data are cited in the main text of this document.
